The article "A Comprehensive Bioinformatic Analysis of NOTCH Pathway Involvement in Stomach Adenocarcinoma" was retracted in 2023. Reasons: suspected computer-generated content; unreliable results or conclusions; concerns about the data; concerns about the results or conclusions.

# A Comprehensive Bioinformatic Analysis of NOTCH Pathway Involvement in Stomach Adenocarcinoma

**DOI:** 10.1155/2021/4739868

**Published:** 2021-12-08

**Authors:** Dongyun Xue, Dong Li, Cong Dou, Junshan Li

**Affiliations:** ^1^Department of Gastroenterology, Shandong Provincial Third Hospital, Cheeloo College of Medicine Affiliated to Shandong University, Jinan City, Shandong Province, China; ^2^Department of Gastroenterology, Zhucheng People's Hospital, Zhucheng, Shandong, China

## Abstract

**Background:**

Activation of NOTCH signaling pathways, which are key regulators of multiple cellular functions, has been frequently implicated in cancer pathogenesis, and NOTCH inhibitors have received much recent focus in the context of cancer therapeutics. However, the role and possible involvement of NOTCH pathways in stomach adenocarcinoma (STAD) are unclear. Here, putative regulatory mechanisms and functions of NOTCH pathways in STAD were investigated.

**Methods:**

Publicly available data from the TCGA-STAD database were utilized to explore the involvement of canonical NOTCH pathways in STAD by analyzing RNA expression levels of NOTCH receptors, ligands, and downstream genes. Statistical analysis of the data pertaining to cancer and noncancerous samples was performed using R software packages and public databases/webservers.

**Results:**

Significant differential gene expression between control and STAD samples was noted for all NOTCH receptors (NOTCH1, 2, 3, and 4), the delta-like NOTCH ligands (DLL-3 and 4), and typical downstream genes (HES1 and HEY1). Four genes (NOTCH1, NOTCH2, NOTCH3, and HEY1) presented prognostic values for the STAD outcome in terms of overall survival. Functional enrichment analysis indicated that NOTCH family genes-strongly correlated genes were mainly enriched in several KEGG signaling pathways such as the PI3K-Akt signaling pathway, human papillomavirus infection, focal adhesion, Rap1 signaling pathway, and ECM-receptor interaction. Gene set enrichment analysis (GSEA) results showed that NOTCH family genes-significantly correlated genes were mainly enriched in four signaling pathways, ECM (extracellular matrix), tumor angiogenesis, inflammatory response, and immune regulation.

**Conclusions:**

NOTCH family genes may play an essential role in the progression of STAD by modulating immune cells and mediating ECM synthesis, angiogenesis, focal adhesion, and PI3K-Akt signaling. Multiple NOTCH family genes are valuable candidate biomarkers or therapeutic targets for the management of STAD.

## 1. Introduction

Gastric cancer is the fifth most common cancer worldwide and a leading cause of cancer-related mortality [1]. Its incidence is particularly high in East Asia and South America [2, 3], translating to high healthcare burden. Despite advances in clinical diagnostic and therapeutic approaches, the majority of gastric cancer patients are first diagnosed at an advanced stage of the disease and recurrence rates are typically high at over 40% [4, 5], suggesting that a substantial need exists for improving molecular diagnostics and therapeutics in stomach cancer. Gastric cancer is subtyped as cardia or noncardia based on its location and distance from the gastroesophageal junction [6] and has a multifactorial etiology and well-recognized risk factors for gastric carcinoma including older age, male gender, genetic susceptibility, *H. pylori* infection, gastroesophageal reflux disease (GERD), and lifestyle factors such as smoking, alcohol, and dietary composition [7, 8]. Among different types, 95% of stomach cancer cases are stomach adenocarcinoma (STAD) [9]. Although substantial research has focused on the etiopathological mechanisms of STAD, the current understanding of tumor mechanisms and regulation remains insufficient [10]. The advent of large multicohort genomic profile repositories of cancer like The Cancer Genome Atlas (TCGA) is facilitating a greater understanding of molecular and genomic aberrations in STAD and their clinical correlates [11, 12].

The NOTCH signaling pathway is an evolutionarily conserved pathway, where NOTCH genes encode a set of transmembrane receptors and 4 type 1 transmembrane NOTCH receptors (NOTCH 1-4) are recognized in mammals, and the NOTCH receptor protein precursor is cleaved in the Golgi apparatus to 2 subunits [13]. NOTCH signaling is essential to several cellular functions and cell behavior necessary for development and homeostasis, including cell proliferation differentiation and death [14, 15]. The role of NOTCH signaling in cancer has been recognized as pleiotropic and its deregulation has been noted in a wide variety of cancers resulting in cancer cell proliferation and reduced cell apoptosis [16–18]. Therefore, NOTCH inhibitors are being investigated as potential anticancer agents [19, 20]. However, effective use of such agents requires molecular characterization of tumors to identify NOTCH pathway activity in specific tumor types and clinical conditions. In the gastric mucosa, NOTCH signaling is implicated in the differentiation process of gastric mucosa and plays a central role in development [21], which later remains essential to maintain the stem cell component by inducing dedifferentiation of gastric epithelial cells into progenitor cells [22]. Consequently, aberrant or continued NOTCH activation in parietal cells has been found to stimulate the development of STAD [22]. In support, evidence from multiple studies indicated that the expression of NOTCH-related genes, NOTCH1, NOTCH2, delta-like 4 (DLL4), and Hes1 is significantly higher in gastric cancer tissue, where NOTCH1, NOTCH2, NOTCH3, and DLL4 were significantly associated with worse tumor characteristics [23]. High expression of NOTCH1, NOTCH3, and Jagged1 has been associated with poor prognosis [24–26]. However, the precise role of NOTCH signaling and ligands in STAD and their relevance to tumor characteristics and molecular mechanisms need further elucidation. In the present study, we aimed to analyze the role of NOTCH signaling in mediating STAD and its clinical characteristics by a comprehensive bioinformatic analysis of publicly available datasets to unravel potential NOTCH-associated mechanisms, correlated genes, and biological pathways.

## 2. Materials and Methods

### 2.1. Study Design of the Current Research

The present research basically followed many previous research investigating the involvement of a specific group of family genes in a specific cancer type by carrying out bioinformatics analyses [27–33]. The flowchart of the present study was displayed briefly as follows: first, the mutation and expression of NOTCH family genes in TCGA-STAD data were investigated. Secondly, survival analysis was performed to research the prognostic value of NOTCH family genes in STAD from the outcome of overall survival and relapse-free survival. Thirdly, the association between clinical variables and prognosis was investigated by performing univariate and multivariate Cox regression analyses. Afterward, the biological functions enriched by the NOTCH family genes-significantly correlated genes were identified by performing the functional enrichment analysis and gene enrichment set analysis. Moreover, the involvement of NOTCH family genes in STAD was investigated by researching the correlation between each NOTCH family gene and tumor-infiltrating immune cells.

### 2.2. cBioPortal Analysis

The cBio Cancer Genomics Portal (cBioPortal) (http://cbioportal.org) was applied to investigate mutations of NOTCH pathway genes in STAD. Queries for visualization and analysis were performed by inputting the information as follows:(1) Cancer type: stomach adenocarcinoma; (2) Six selected studies: Stomach Adenocarcinoma (Pfizer and UHK, Nat Genet 2014, 100 samples), Stomach Adenocarcinoma (TCGA, Firehose Legacy, 478 samples), Stomach Adenocarcinoma (TCGA, Nature 2014, 295 samples), Stomach Adenocarcinoma (TCGA, PanCancer Atlas, 440 samples); Stomach Adenocarcinoma (U Tokyo, Nat Genet 2014, 30 samples), and Stomach Adenocarcinoma (UHK, Nat Genet 2011, 22 samples); (3) Molecular profiles: Mutations, Structural variants, and copy number alterations; (4) Select Patient/Case Set: all samples (1365); and (5) Enter Genes: NOTCH1, NOTCH2, NOTCH3, NOTCH4, DLL1, DLL3, DLL4, JAG1, JAG2, HES1, and HEY1. After the queries were submitted, tracks were added including the study of origin, mutation spectrum, mutation count, overall survival status, overall survival (months), disease-free status, and disease-free period (months). Next, the cancer type summary of six included cancer studies regarding STAD was visualized based on filtering.

### 2.3. The Dysregulation of NOTCH Family Genes in STAD

Level 3 HT-seq data of STAD patients with the fragments per kilobase per million (FPKM) format were downloaded from the TCGA database. Samples without clinical information were removed, and 407 samples containing 375 STAD tumor samples and 32 healthy control samples were included for the subsequent analysis. The mRNA expression levels of NOTCH family genes in STAD were analyzed and visualized using the “ggplot” package (version 3.3.3) in R (version 3.6.3).

### 2.4. Survival Analysis

Kaplan-Meier analysis was performed to compare survival rates between “high” and “low” expression groups of each NOTCH family genes. The Kaplan-Meier curves were plotted using the KM plotter web tool (URL: https://kmplot.com/analysis/). Patients were divided into two groups based on the median gene expression value, and log-rank tests (*p*[LogRank]) were used to compare the survival between the “high-” expression group (red line) and “low-” expression groups (blue line). Two types of prognostic parameters were analyzed, including overall survival (OS) and disease-specific survival (DSF).

### 2.5. Association of Metadata Variables for the TCGA-STAD Data with NOTCH Gene Expression Levels

The subsequent analysis was based on the TCGA-STAD dataset, which included 407 samples containing 375 STAD tumor samples and 32 healthy control samples. The mRNA expression levels of each gene within 11 NOTCH family genes and clinicopathological details were documented, and general metadata information pertaining to STAD samples was obtained. Data analysis was performed using R (version 3.6.3). Based on the median value of the expression level of each NOTCH family gene, the STAD samples were divided into two groups, a “low-” expression group of and a “high-” expression group.

### 2.6. Univariate and Multivariate Cox Regression Analyses

The association between clinical variables and prognosis was investigated by performing univariate and multivariate Cox regression analyses. The “coxph” function in the R “survival” package (version 3.2-10) was applied and the cox regression module was used. Overall survival was selected as the prognostic outcome type. The clinical variables included in the analysis were T stage, N stage, M stage, age, gender, race, pathologic stage, primary therapy outcome, residual tumor, reflux history, histologic grade, antireflux treatment, *H. pylori* infection, and expression level of each NOTCH family gene.

### 2.7. Forest Plots

Based on the results (HR, 95% CI, *p* value) obtained by univariate and multivariate cox regression analyses, two forest plots were plotted using the “ggplot2” package (version 3.3.3) in R (version 3.6.3). The HR (hazard ratio) can be considered to represent a relative risk of death that compares one instance of a binary feature to the other instance-reference category. Thus, an HR > 1 indicates an increased risk of death, while an HR < 1 represents a decreased risk of death.

### 2.8. ROC Curve Analysis to Evaluate the Diagnostic Value of NOTCH Family Gene Expression

ROC curve analysis for each NOTCH family gene expression data was conducted by using the “pROC” package (version 1.17.0.1) and visualized using “ggplot2” package (version 3.3.3). The predicted outcome parameter was defined as clinical status (STAD tumor vs. normal). In the ROC analysis, the *x*-axis represents the false-positive rate (FPR), and the *y*-axis represents the true-positive rate (TPR).

### 2.9. Identification of Significantly Correlated Genes of NOTCH Family Genes

As initial analysis indicated nonsignificant deregulation of DDL1 in STAD, genes correlated with the remaining NOTCH family genes were used for functional enrichment analysis and GSEA. Analysis was performed using the “stat” package (version 3.6.3) in R (version 3.6.3). The Pearson correlation test, a parametric correlation test that measures a linear relationship between the two groups, was applied. Only protein coding genes were retained. According to the conventional approach to interpret the correlation coefficient, the correlation coefficient “*r*” value with 0.90–1.00 was very strong correlation, 0.70–0.89 indicated strong correlation, 0.40–0.69 represented moderate correlation, 0.10–0.39 indicated weak correlation, and 0.00–0.10 should be interpreted with negligible correlation [34]. Overlapping genes among individual NOTCH family genes' significantly strongly correlated genes were identified and used for the subsequent analysis.

### 2.10. Functional Enrichment Analysis of Significantly Strongly Correlated Genes of NOTCH Family Genes

Overlapping genes among the 10 NOTCH family genes-correlated genes with |cor_pearson | >0.7 and *p*_pearson < 0.001 identified previously were used for the functional enrichment analysis to identify significantly enriched functional terms. The gene names were converted to the Entrez ID by using the “https://bioconductor.org/packages/release/data/annotation/html/org.Hs.eg.db.html” package (version 3.10.0) in R (version 3.6.3). Functional enrichment analysis was performed by using the “clusterProfiler” package (version 3.14.3) in R (version 3.6.3). GO terms including BP (biological process), CC (cellular component), MF (molecular function), and KEGG pathways that were significantly enriched by the correlated genes were identified at a threshold of *p*.adj < 0.05 and *q* value < 0.2. Bubble charts were plotted to visualize the functional enrichment results using the ggplot2 package (version 3.3.3).

### 2.11. Gene Set Enrichment Analysis

The differentially expressed genes (DEGs) between STAD samples and healthy control samples from the TCGA-STAD dataset were identified by using “DESeq2” (version 1.26.0) in R (version 3.6.3). As GSEA can have higher accuracy when more genes are included, the threshold for defining significantly correlated genes was set at ∣cor_pearson | >0.4 and *p*_pearson < 0.001 and these genes were then used for GSEA. The log_2_FC (fold change) values of the 10 NOTCH family genes-significantly correlated genes were obtained and used for the gene set enrichment analysis (GSEA). GSEA analysis was performed using the “clusterProfiler” package (version 3.14.3) in R (version 3.6.3). The functional terms satisfying a threshold of normalized enrichment score ∣NES | >1, nominal *p* value (NOM *p* value) < 0.05, and a false discovery rate (FDR) *q* value < 0.25 were considered as significantly enriched terms.

### 2.12. Gene-Gene Interaction (GGI) Network Analysis

GeneMANIA (URL: http://genemania.org; accessed on 1^st^ October 2021) was used to construct the gene-gene interaction network (GGI). All 11 NOTCH family genes were used as the input, and two functions, NOTCH signaling pathway and regulation of the NOTCH signaling pathway, were selected. The GGI network was constructed by an automatically selected weighting method and downloaded.

### 2.13. Correlation of Each NOTCH Family Gene Expression with Immune Cells in STAD

The correlation of each NOTCH family gene with immune cells in STAD tumor samples was investigated by using Pearson's test performed by using “GSVA” package (version 1.34.0) in R (version 3.6.3). The “ssGSEA” algorithm, a built-in algorithm in the “GSVA” package, was used for statistical analysis. 24 tumor immune infiltration cells (TIICs) were analyzed, which included aDC (activated DC), B cells, CD8 T cells, cytotoxic cells, DC, eosinophils, iDC (immature DC), macrophages, mast cells, neutrophils, NK CD56bright cells, NK CD56dim cells, NK cells, pDC (plasmacytoid DC), T cells, T helper cells, Tcm (T central memory), Tem (T effector memory), Tfh (T follicular helper), Tgd (T gamma delta), Th1 cells, Th17 cells, Th2 cells, and Treg cells. The gene markers of the 24 TIICs were obtained from a previously published study. A lollipop plot was used to illustrate the correlation of each NOTCH family gene expression level with the 24 TIICs in STAD samples.

## 3. Results

### 3.1. NOTCH Family Gene Alterations and mRNA Expression in STAD

The cBioPortal online tool was used to analyze the gene expression of NOTCH family member genes in STAD patients. NOTCH gene alterations in STAD ranged from 1.6% to 9% (Figure 1(a)). The structural variant data, mutation data, and CNA (copy number alteration) data from 6 studies are depicted in Figure 1(b).

The analysis of 375 STAD tumor samples and 32 healthy control samples (Figure 1(c)) showed significant overexpression of 10 genes (NOTCH1, NOTCH2, NOTCH3, NOTCH4, DLL1, DLL4, JAG1, JAG2, HES1, and HEY1) in STAD tumor samples compared with healthy control samples, whereas the expression of DDL1 was not significantly different between control and cancer samples. Analysis of 27 STAD tumor samples and 27 healthy control samples (Figure 1(d)) showed that 9 genes (NOTCH1, NOTCH3, NOTCH4, DLL4, JAG1, JAG2, HES1, and HEY1) were significantly upregulated in STAD tumor samples compared with healthy control samples, whereas 2 genes' (NOTCH2 and DDL1) expression levels did not differ significantly.

### 3.2. Prognostic Values of NOTCH Family Genes in STAD

Four genes (NOTCH1, NOTCH2, NOTCH3, and HEY1) were found to be significantly associated with overall survival in STAD, whereas the remaining 7 NOTCH genes (NOTCH4, DLL1, DLL3, DLL4, JAG1, JAG2, and HES1) did not display a prognostic value for overall survival (Figure 2). The upregulation of 3 genes (NOTCH2, NOTCH3, and HEY1) indicated significantly worse overall survival outcome while the upregulation of NOTCH1 indicated better overall survival outcome. 3 genes (NOTCH1, NOTCH3, and DLL3) were found significantly correlated with relapse-free survival in STAD, while the remaining 8 genes (NOTCH2, NOTCH4, DLL1, DLL4, JAG1, JAG2, HES1, and HEY1) have no prognostic value (Figure 3).

### 3.3. Metadata Variables of TCGA-STAD Patients Associated with NOTCH Gene Expression

The clinical metadata and gene expression data of 375 primary STAD tumor samples were downloaded from the TCGA database (Table S1). None of the metadata variables were found significantly related with the expression level of NOTCH1. For NOTCH2 gene expression, 3 clinical variables, T stage (*p* = 0.001), race (*p* = 0.001), and OS event (*p* = 0.038) were found statistically significantly related. For N0TCH3 gene expression, 3 clinical variables, T stage (*p* = 0.039), pathologic stage (*p* = 0.049), and PFI event (*p* = 0.013), were significantly related to expression. Two clinical variables, anatomic neoplasm subdivision (*p* = 0.046) and OS event (*p* = 0.022), were statistically significantly related to the expression levels of NOTCH4. Two clinical variables, histological type (*p* = 0.040) and anatomic neoplasm subdivision (*p* = 0.039), were significantly related to the expression levels of the DLL1 gene, and two clinical variables, DSS event (*p* = 0.039) and PFI event (*p* = 0.013), were statistically significantly related to the expression levels of the DLL3 gene. For the DLL4 gene, only 1 clinical variable, anatomic neoplasm subdivision (*p* < 0.001), was statistically significantly associated. One clinical variable, T stage, was statistically significantly associated with the expression of the JAG1 gene, while no variables were associated with the JAG2 gene. Three clinical variables, race (*p* = 0.017), histological type (*p* = 0.010), and histologic grade (*p* = 0.018), were found to be significantly related to HES1 expression, while no clinical variable was significantly associated with the expression of HEY1.

### 3.4. Univariate and Multivariate Cox Regression Analyses

Table S2 shows the results of univariate and multivariate cox regression analyses. The univariate analysis showed that multiple clinical variables, T stage (*p* = 0.011), N stage (*p* = 0.002), M stage (*p* = 0.004), age (*p* = 0.005), pathologic stage (*p* < 0.001), primary therapy outcome (*p* < 0.001), and residual tumor (*p* < 0.001), were statistically significantly related to the overall survival of STAD patients; while the remaining clinical variables, gender, race, reflux history, histologic grade, antireflux treatment, H pylori infection, and gene expression levels of NOTCH1, NOTCH2, NOTCH3, DLL1, DLL3, DLL4, JAG1, JAG2, HES1, and HEY1, were not significantly associated with the overall survival. The multivariate analysis results showed that two clinical variables, age (*p* = 0.025) and primary therapy outcome (*p* < 0.001), were significantly associated with overall survival whereas the other variables, T stage, N stage, M stage, pathologic stage, residual tumor, NOTCH2 gene expression, and NOTCH4 gene expression, were not significantly associated.

### 3.5. Forest Plot Visualization

The univariate Cox regression analysis indicated that several factors, higher T stage (T3 & T4) (*p* = 0.011), higher N stage (N1 & N2 & N3) (*p* = 0.002), M stage (M1) (*p* = 0.004), age (>65) (*p* = 0.005), higher pathologic stage (stage III & stage IV) (*p* < 0.001), primary therapy outcome (PD & SD) (*p* < 0.001), and residual tumor (R1 & R2) (*p* < 0.001), were negative predictors for overall survival outcome in STAD (Figure 4(a)).  Figure 4(b) shows the results of the multivariate cox regression analysis, indicating that the factors age (>65) (*p* = 0.025) and primary therapy outcome (PD & SD) (*p* < 0.001) were negative predictors for overall survival outcome.

### 3.6. Diagnostic Value of NOTCH Family Gene Expression in STAD

The diagnostic value of each NOTCH family gene expression by the ROC curve was evaluated.  Figure 5 shows that the majority of NOTCH family genes' expression showed moderate accuracy in discriminating STAD versus control (NOTCH1: AUC = 0.739; NOTCH3: AUC = 0.804; NOTCH4: ACU = 0.833; DLL4: AUC = 0.891; JAG1: AUC = 0.766; JAG2: AUC = 0.846; HES1: AUC = 0.754; and HEY1: AUC = 0.792). The AUC values of the remaining three genes (NOTCH2: AUC = 0.641; DLL1: AUC = 0.547; and DLL3: AUC = 0.682) were less than 0.7, indicating a low diagnostic value.

### 3.7. Biological Functions of Significantly Correlated Genes of NOTCH Family Genes

By selecting the significantly strongly correlated genes of each NOTCH family gene, 163 genes were obtained.  Figure 6 depicts bubble charts for 3 GO terms and KEGG pathways enriched by these 165 genes.

NOTCH family genes-strongly correlated genes were mainly enriched in several biological processes (e.g., regulation of angiogenesis, extracellular matrix organization, and endothelial cell proliferation) (Figure 6(a) and Table S3), several cellular components (e.g., collagen-containing extracellular matrix, cell-substrate adherens junction, and focal adhesion) (Figure 6(b) and Table S4), several molecular functions (e.g., extracellular matrix structural constituent, growth factor binding, cytokine binding, and collagen binding) (Figure 6(c) and Table S5), and several KEGG pathways (e.g., PI3K-Akt signaling pathway, human papillomavirus infection, focal adhesion, Rap1 signaling pathway, and ECM-receptor interaction) (Figure 6(d) and Table S6).

### 3.8. Results of GSEA Analysis

The results of GSEA of the NOTCH family genes-significantly correlated genes are shown in Table S7. Some of the terms of interest are visualized in Figure 7. It was evident that these genes were mainly enriched in four signaling pathways, ECM- (extracellular matrix-) related pathways (e.g., collagen biosynthesis and modifying enzymes, ECM proteoglycans, syndecan 1 pathway, integrin cell surface interactions, and focal adhesion-PI3K/AKT/MTOR signaling pathway) (Figure 7(a)), tumor angiogenesis-related pathways (e.g., signaling by PDGF, platelet aggregation plug formation, and vascular smooth muscle contraction) (Figure 7(b)), inflammatory response (e.g., inflammatory response pathway, and cytokine-cytokine receptor interaction) (Figure 7(c)), and immune regulation (e.g., immunoregulatory interactions between a lymphoid and a nonlymphoid cell and the human complement system) (Figure 7(d)).

### 3.9. Visualization of Gene-Gene Interaction (GGI) Network

Figure 8 shows 20 genes which were potentially frequently interacting with the 11 NOTCH family genes. These 20 interacting genes include DLK1, MAML1, DNER, APH1B, PSENEN, APH1A, MFNG, DTX1, LFNG, NOTCH2NLR, NOTCH2NLA, GNPTAB, MIB1, POFUT1, NCSTN, SNED1, ADAM10, RBPJ, HEG1, and DLK2.

### 3.10. Correlation of NOTCH Family Gene Expression and Immune Cells in STAD

Figure 9 shows the correlation between NOTCH family gene expression and immune cells in STAD. NOTCH1 gene expression was positively correlated with many TIICs including Tem, Tcm, NK cells, TFH, eosinophils, NK CD56dim cells, T helper cells, Th2 cells, and Th1 cells. NOTCH2 gene expression was positively correlated with majority of TIICs (Tem, Tcm, NK cells, macrophages, eosinophils, mast cells, iDC, DC, Th1 cells, TFH, T cells, T helper cells, CD8 T cells, B cells, cytotoxic cells, neutrophils, Treg cells, aDC, Tgd, and NK CD56dim cells) but negatively correlated with Th17 cells.

## 4. Discussion

Overall, the comprehensive bioinformatic analysis demonstrated that NOTCH family genes are likely to play key roles in STAD pathogenesis via the mechanisms of immune cell modulation, mediating epithelial-mesenchymal transformation (EMT), angiogenesis, focal adhesion, and PI3K-Akt signaling. Except DDL1, significant overexpression of NOTCH genes in STAD tissue was noted, supporting the notion that activation of NOTCH signaling plays a mechanistic role in STAD. Survival analysis showed that NOTCH2, NOTCH3, and HEY1 predicted worse overall survival. A role of NOTCH signaling in immune escape via NOTCH3 upregulation has been documented, associated with lower antitumor activity of CD8+ T cells and greater infiltration of immune suppressive Treg and M2 macrophages, with upregulation of immune checkpoint genes, suggesting that NOTCH3 expression may be a useful biomarker and enable the prediction of response to immune checkpoint blockers [35]. A very high frequency of NOTCH2 expression with nuclear translocation (97.3%) has been documented in gastric cancer versus noncancerous mucosal tissue (10%) [36]. Others have shown that NOTCH2 possessed a tumor suppressor function in gastric cancer by modulation of the PI3K/Akt pathway and MMP9 suggesting the importance of physiological levels of NOTCH2 expression in preventing stomach carcinogenesis [37], supported by another report of higher NOTCH2 expression in early-stage gastric tumors as compared to advance-stage tumors [38]. These inconsistencies highlight the pleiotropic role of NOTCH signaling and receptors in cancer, whereby they may produce pro- or antioncogenic effects on different and even on the same tumor at different times [39, 40]. The transcriptional repressor HEY1 gene is a NOTCH target signal transducer [41] and its overexpression has been found to promote gastric cancer [42].

In the present analysis, NOTCH1 upregulation was found to indicate better overall and relapse-free survival, which was aligned with a previous finding of high NOTCH1 expression in early-stage gastric cancer and the association with improved survival outcome in this subtype [43]. In contrast, NOTCH1 activation has been found to indicate worse prognosis in gastric cancer [44–46], while some have noted that high NOTCH1 was linked to worse prognosis in intestinal-type gastric cancer alone [47]. A meta-analysis [23] showed that high NOTCH1 expression was linked to several adverse clinical variables in gastric cancer including a larger size, noncardia location, lymphovascular invasion, and metastasis. Mechanistically, activation of NOTCH1 signaling has been found to mediate gastric cancer progression via the cyclooxygenase 2 pathway [48]. In addition, NOTCH1 signaling has been implicated in promoting EMT and proliferation of gastric epithelial cells [35], apart from promoting gastric cancer via its interaction with STAT3 and TWIST [45]. However, another report has also validated an antitumor role of NOTCH1 activation, showing low expression in gastric cancer tumor tissue, aligned with the present finding [48]. In case of lung cancer, opposing effects of NOTCH1 activation have been recognized in lung adenocarcinoma versus lung squamous cell cancer and attributed to differences in the NOTCH1-interacting or coexpressed proteins [49].

The negative NOTCH regulator delta-like canonical Notch ligand 3 (DLL3) predicted relapse-free survival in STAD and has attracted recent attention as a novel cancer target due to its role in multiple neuroendocrine cancers [50], with the advent of DDL3-targeting agents such as antitumor drug-antibody conjugate Rova-T and AMG-19 [51, 52]. Here, the highest gene aberration rate was found for NOTCH2, supported by a previous report, which analyzed NOTCH gene mutation rates in the TCGA data using cBioPortal and reported the highest gene mutation rate for NOTCH2 and NOTCH3 [41]. Consistently, the present analysis found that NOTCH2 and NOTCH3 significantly predicted 3 clinical variables each including the tumor stage. However, the Cox regression analysis, which allows the analysis of multiple predictors unlike Kaplan-Meier analysis, did not indicate significant hazard ratios for any of the NOTCH genes for survival in STAD, possibly reflecting the time- and context-dependent role of NOTCH signaling in the pathogenesis of STAD. When considering the discriminant value of NOTCH genes for STAD versus the healthy state, significantly, a moderate diagnostic accuracy was evident for most genes, with DLL4 showing the highest AUC value (0.891). The activation of DLL4-mediated NOTCH signaling is associated with angiogenesis and has been shown to stimulate MMP2 proenzyme expression and promote gastric carcinogenesis [53]. Furthermore, the potential of anti DLL4 treatment, which has been shown to inhibit tumorigenesis by restricting tumor vasculature has been shown in gastric cancer [54, 55].

The most significant biological processes enriched by NOTCH genes-strongly correlated genes in STAD included regulation of tumor cell, migration, angiogenesis, extracellular matrix organization, and endothelial cell proliferation. During invasion, individual tumor cells exhibit two main different modes of migration, leading to metastasis [56]. The top biological process enriched was amoeboid-type migration, suggesting that NOTCH signaling appears to be associated with an amoeboid-type migration strategy of cancer cell motility in STAD, which is marked by distinct interactions with the surrounding tumor microenvironment [56]. In tandem, the top cellular components and molecular functions enriched included cell-cell junctions, cell-substrate junction, and extracellular matrix, cell adhesion molecule, and growth factor binding. Cell adhesion molecules play a key role in tumor metastasis and immune cell recruitment, and canonical NOTCH signaling is known to promote cell adhesion via the expression of integrins and related cell adhesion molecules, while the role of noncanonical NOTCH signaling in cell adhesion is not well elucidated [57, 58]. The role of NOTCH signaling in tumor angiogenesis by multiple mechanisms has been described, mediated chiefly by the ligands DLL4 and Jagged1, whereby DLL4 inhibits neoangiogenesis while competitive binding of Jagged1 is promoted [59]. NOTCH signaling is an essential component of the cellular crosstalk within the tumor microenvironment by juxtacrine signaling between NOTCH receptors and ligands, interacting with other pathways including Wnt, thus regulating cancer stem cell renewal, angiogenesis, and immune functions [60]. The KEGG pathway analysis showed that NOTCH genes-strongly correlated genes were most significantly enriched in the PI3K/Akt pathway in STAD. The PI3K/Akt pathway has been chiefly implicated in tumor metastasis and chemotherapy resistance, and PIK3CA is a well-recognized oncogene whose mutations are associated with gastric cancer [61, 62]. Furthermore, a synergistic effect of NOTCH1 and PI3K/Akt inhibition on restricting gastric cancer has been reported [63]. These findings are corroborated by an earlier report analyzing gastric cancer immune microenvironment-related competitive endogenous RNAs that also found PI3K/Akt and human papillomavirus KEGG pathways as significantly enriched [64]. An oncogenic role of human papilloma virus infection in gastric adenocarcinoma was reported, where 29% lesions showed HPV-16 DNA [65], although the association has not been consistently found. Overall, the functional enrichment and GSEA results were largely corroborative.

Immune infiltration and antitumor immune evasion are a key mechanism of tumor progression. Effector memory T cells (Tem) and central memory T cells (Tcm) were highly correlated with NOTCH1, NOTCH2, NOTCH3, DLL1, and DLL4 gene expression in STAD. Memory T cell subsets reflect immune response to tumor antigens and have been found to be indicators of the stage and clinical characteristics of gastric cancer [65]. NOTCH1 signaling is known to regulate CD8+ T cell responses, increasing differentiation to effector T cells and maintenance of memory T cells, thereby regulating immune surveillance and tumor suppression [66]. NOTCH2 signaling is needed to generate antitumor cytotoxic T cell responses [67]. Possibly, therapeutic agonistic modulation of NOTCH signaling could serve as an antitumor effector T-cell immune modulator and improve the efficacy of immunotherapy in STAD [68, 69]. NOTCH2 and NOTCH3 expression was inversely linked to Th17 cells in STAD. Increased tumor-infiltrating CD4+ Th17 cells and proinflammatory IL-17 is noted in gastric cancer and associated with tumor progression [70]. The advent of adaptive T cell-based tumor therapies such as chimeric antigen receptor T cell therapy may be a promising modality in STAD, and a deeper understanding of NOTCH signaling in this context could enable improved treatment strategies.

These findings must be viewed in light of the limitations of the present study, whereby *in vitro* or *in vivo* experiments were not performed for experimental validation of the identified role of NOTCH signaling in STAD, which should be attempted in future studies. Furthermore, the value of specific NOTCH-targeting drugs and ligands [20] in STAD merits deeper investigation considering the present findings. Most importantly, these data also suggest the potential utility of molecular characterization of STAD patient subgroups amenable to therapy with selective NOTCH ligands as a precision medicine approach.

## 5. Conclusion

Comprehensive bioinformatics analysis of NOTCH signaling-related genes in STAD indicated that NOTCH activation is a key participant in mediating the development and progression of STAD via multiple pathways including immune cell modulation, mediating ECM synthesis, angiogenesis, focal adhesion, and regulation PI3K-Akt signaling. Upregulated NOTCH2, NOTCH3, and HEY1 were associated with worse survival prognosis whereas NOTCH1 indicated improved survival and multiple NOTCH family gene expression showed a moderate diagnostic biomarker value for STAD.

## Figures and Tables

**Figure 1:** Alteration frequency and aberrant expression of the NOTCH family genes in STAD. (a) The mRNA expression (RNA Seq V2 RSEM) of the NOTCH pathway family genes in STAD. (b) The summary of the cancer types in the cBioPortal was used to calculate the percentages of STAD cases of the NOTCH family genes. (c) The mRNA level of NOTCH family genes between STAD tissues and unpaired normal oral tissues in TCGA. (d) The mRNA expression level of NOTCH family genes in STAD tissues and paired normal oral tissues in TCGA. ns: not significant (*p* ≥ 0.05); ^∗^*p* < 0.05; ^∗∗^*p* < 0.01; ^∗∗∗^*p* < 0.001.

**Figure 2:** Survival analysis results for OS (overall survival) by using KM plots web tool.

**Figure 3:** Survival analysis results for RFS (relapse-free survival) using KM plots web tool.

**Figure 4:** The forest plots showing the outcome of univariate and multivariate Cox regression analyses with NOTCH family genes and other clinicopathologic parameters as predictors and overall survival (OS) in STAD patients as outcome. (a) The forest plot showing the results of univariate regression analysis. (b) The forest plot showing the results of the multivariate regression analysis.

**Figure 5:** ROC curves for NOTCH family genes in healthy control tissue and STAD.

**Figure 6:** Functional enrichment analysis results of the significantly strongly correlated genes of NOTCH family genes. (a) GO term BP (biological process); (b) GO term CC (cellular component); (c) GO term MF (molecular function); (d) KEGG pathways. In the bubble charts, the bubble size is consistent with the number of gene counts enriched in a specific term. The depth of the bubble color is consistent with the *p*.adj value. The darker the bubble color, the smaller the *p* adjustment value, indicating that the specific functional term is more significantly enriched.

**Figure 7:** The results of the GSEA showing that NOTCH family genes-significantly correlated genes were mainly enriched in four signaling pathways, ECM (extracellular matrix) (a), tumor angiogenesis (b), inflammatory response (c), and immune regulation (d).

**Figure 8:** The GGI network consisted of the 11 NOTCH family genes.

**Figure 9:** Lollipop plot showing the correlation between each NOTCH family gene expression and 24 TIICs in STAD. In the color bar, the darker the color, the smaller the *p* value, indicating higher statistical significance. The bubble size represents the correlation value, and the bigger the bubble size, the greater the correlation value.

## Data Availability

The data analyzed during the current study are available in the TCGA database with the accession number TCGA-STAD. The original contributions presented in the study are included in the article; further inquiries can be directed to the corresponding author.

## Supplementary Materials

Supplementary Materials Table S1: association of clinical characteristics of the TCGA-OSCC patients with the expression level of the DEFB1 gene. Table S2: risk assessment of NOTCH components on overall survival of STAD patients, analyzed by univariate and multivariate Cox regression. Table S3: the top 20 GO term biological processes (BP), enriched by the NOTCH family genes-strongly correlated genes. Table S4: the top 20 GO term cellular components (CC), enriched by the NOTCH family genes-strongly correlated genes. Table S5: the top 20 GO term molecular functions (MF), enriched by the NOTCH family genes-strongly correlated genes. Table S6: the top 20 KEGG signaling pathways, enriched by the NOTCH family genes-strongly correlated genes. Table S7: results of the GSEA analysis based on the NOTCH family genes-significantly correlated genes.
